# Circ_0058792 regulates osteogenic differentiation through miR-181a-5p/Smad7 axis in steroid-induced osteonecrosis of the femoral head

**DOI:** 10.1080/21655979.2022.2074617

**Published:** 2022-05-25

**Authors:** Ning Han, Fei Qian, Xianping Niu, Guoting Chen

**Affiliations:** a Department of Orthopaedic Traumatology, Shanghai East Hospital, Tongji University School of Medicine, Shanghai, China; b Department of Stomatology, Shanghai East Hospital, Tongji University School of Medicine, Shanghai, China; c Department of Geriatric Medicine, Shanghai East Hospital, Tongji University School of Medicine, Shanghai, China; d Department of Emergency Traumatology, Shanghai East Hospital, Tongji University School of Medicine, Shanghai, China

**Keywords:** Steroid-induced ONFH, circ_0058792, miR-181a-5p, osteogenic differentiation, Smad7

## Abstract

Osteonecrosis of the femoral head (ONFH) caused by steroids is a severe orthopedic disorder resulting from the use of high-dose steroid drugs, characterized by structural changes in the bone, joint dysfunction, and femoral head collapse. CircRNAs and miRNAs have increasingly been suggested to play pivotal roles in osteogenic differentiation and osteogenesis. Significant upregulation of circ_0058792 was observed in patients with steroid-induced ONFH. Bioinformatic analysis showed that circ_0058792 might act as a sponge for miR-181a-5p. This study further investigated the mechanisms underlying the role of circ_0058792 and miR-181a-5p in osteogenic differentiation in methylprednisolone-induced ONFH rats and MC3T3-E1 cells. The results showed a notable decrease in the serum of miR-181a-5p in methylprednisolone-induced ONFH rats. Silencing of circ_0058792 using siRNAs and overexpression of miR-181a-5p significantly increased alkaline phosphatase activity and matrix mineralization capacity. Additionally, markers for osteogenic differentiation were significantly upregulated in miR-181a-5p-transfected cells. However, overexpression of circ_0058792 and the addition of the miR-181a-5p inhibitor reversed this increase. Smad7 was identified to be miR-181a-5p’s direct target and circ_0058792 was confirmed to be miR-181a-5p’s competing endogenous RNA (ceRNA). Upregulation of miR-181a-5p promotes phosphorylation of Smad2 and Smad3. Furthermore, circ_0058792 and miR-181a-5p had opposing effects on Smad7 expression. Collectively, these findings indicate that circ_0058792 regulates osteogenic differentiation by sponging miR-181a-5p via the TGF-β/Smad7 pathway. These findings elucidated the functions of circ_0058792 and miR-181a-5p in the regulation of steroid-induced ONFH. Our findings also indicated that circ_0058792 and miR-181a-5p are possible diagnostic markers and therapeutic targets for treating steroid-induced ONFH.

## Highlights

- Circ_0058792 was significantly upregulated in steroid-induced ONFH patients.
- MiR-181a-5p was markedly downregulated in steroid-induced ONFH rats.
- Circ_0058792 and miR-181a-5p play important roles in the development of ONFH.
- Circ_0058792 sponging miR-181a-5p regulated the TGF-β/Smad7 pathway.

## 1. Introduction

Osteonecrosis of the femoral head (ONFH), a frequently occurring bone disorder, is a progressive and disabling chronic disease that can cause femoral head collapse, finally leading to total hip arthroplasty [1]. ONFH can generally be divided into two groups: non-traumatic and traumatic. Of these, steroid-mediated ONFH is a frequent non-traumatic subtype, which is on the rise and has become the first pathogenesis of ONFH [2]. However, long-term use of steroids in some patients may increase the incidence of steroid-induced ONFH, which significantly decreases their quality of life. Presently, as far as we know, the exact pathogenesis of steroid-induced ONFH remains unclear; however, several hypotheses have been proposed, including lipid metabolism disorder [3], intravascular coagulation [4], inflammation, cell apoptosis [5], and decreased osteogenic potential of bone marrow stem cells (BMSCs) [2,6].

CircRNAs are closed-loop, covalent, non-coding RNAs (ncRNAs) with the absence of a 5′ cap structure and 3′ polyA tail [7,8]. CircRNAs have been frequently suggested to be related to cell homeostasis, which plays a pivotal role in some physiological processes [9]. To date, the specific mechanism of circRNAs is the miRNA sponge or competing endogenous RNA (ceRNA) mechanism [10]. MicroRNAs (miRNAs) are small endogenous ncRNAs that are 21–25 nucleotides (nt) in length and can specifically recognize the complementary 3′ UTR region of target mRNA, preventing protein translation or promoting target mRNA degradation [11,12]. CircRNAs and miRNAs play important roles in regulating post-transcriptional gene expression. In the human genome, miRNAs regulate approximately 30% of genes that encode proteins [13]. The expression of circRNAs and miRNAs is tissue-specific, and many of them are highly evolutionary conserved [7]. Accumulating evidence suggests that circRNAs and miRNAs can be used as biomarkers and diagnostic tools for diseases such as cancer, infections, nervous system disorders, cardiovascular disorders, osteoporosis, and diabetes [14,15].

Numerous studies have suggested that miRNAs and circRNAs play key roles in the regulation, proliferation, and differentiation of osteoblasts, and their dysregulation is related to steroid-mediated ONFH [16,17]. Chen *et al*. demonstrated that the upregulated circRNA, CDR1as, was involved in osteogenic/adipogenic differentiation disorder by regulating the miR-7-5p/WNT5B axis in steroid-induced BMSCs [18]. Using a miRNA microarray, Li *et al*. found that 11 miRNAs were differentially expressed (9 down-regulated and 2 up-regulated) between the healthy and patient (systemic lupus erythematosus (SLE) and steroid-mediated ONFH, SLE-SONFH) groups [16]. A study based on qRT-PCR and miRNA microarray revealed that miR-335 and miR-132-3p were upregulated; however, let-7c-1-3p and miR-466b-2-3p were downregulated in femoral head BMECs of methylprednisolone-induced rats, a commonly used steroid-induced ONFH model [19]. Wang *et al*. demonstrated that miR-516b-5p, miR-647, miR-452-3p, and miR-601 were markedly upregulated, whereas miR-122-3p expression was markedly decreased in BMSCs of SONFH cases relative to normal subjects [17]. The upregulation of miR-132-3p markedly suppresses MC3T3-E1 cell growth and differentiation [20]. These findings demonstrated that circRNAs and miRNAs can serve as novel biomarkers or therapeutic targets for steroid-induced ONFH.

In a recent study, we identified a series of differentially expressed circRNAs derived from BMSCs of patients with steroid-induced ONFH using a microarray analysis technique. A variety of upregulated or downregulated circRNAs were verified using qRT-PCR (data not shown). We confirmed that circ_0058792 was markedly upregulated compared with that in healthy individuals. However, the function of circ_0058792 in ONFH development has not yet been investigated. We verified that circ_0058792 could sponge miR-181a-5p to eliminate miR-181a-5p’s modulation. In several previous studies, miR-181a-5p was recognized as an essential regulator of various diseases, including acute pancreatitis [21], high-fat-induced hyperglucagonemia [22], vascular inflammation, and atherosclerosis [23]. Recently, a study discovered that miR-181a-5p was significantly downregulated in patients with SEL-steroid-induced ONFH compared to that of the SEL controls [24].

This study aimed to explore the specific mechanisms of circ_0058792 and miR-18a-5p in the development of steroid-induced ONFH and differentiation of osteoblasts. The effects of circ_0058792 and miR-181a-5p on osteogenic differentiation were investigated in MC3T3-E1 cells. The downstream target proteins were identified using a dual-luciferase assay. Our results demonstrate that the potential circ_0058792/miR-181a-5p/Smad7 axis might be related to steroid-induced ONFH occurrence. Thus, circ_0058792 and miR-181a-5p could be used as novel therapeutic targets for the treatment of steroid-induced ONFH.

## 2. Materials and methods

### 2.1 Establishment of the steroid-induced ONFH rat model

Sprague-Dawley (SD) female rats weighing 190–220 g were obtained from the Academy of Military Medical Sciences (Beijing, China) and raised in a standard environment at 24 ± 2°C and 12 h/12 h light-dark cycle conditions. All animals were permitted to eat food and drink water *ad libitum*. Each experiment was carried out in accordance with the laboratory animal use guidelines approved by the Animal Care Committee of China. The study protocol was approved by the Experimental Animal Center of the Shanghai East Hospital (No. 2021–0015).

This study randomized the animals into two groups, with 10 animals in each group, including the control and methylprednisolone sodium succinate (Sinopharm, China) groups. We initially administered lipopolysaccharide (LPS) intraperitoneally (Sigma-Aldrich, Shanghai, China) to rats in the methylprednisolone group at 20 μg/kg body weight (BW) for a 2-day period, followed by intramuscular injection of methylprednisolone at 40 mg/kg BW at 24 h intervals for a 3-day period [25]. Equivalent amounts of saline were administered to control rats. The rats were raised continuously for four weeks under these conditions.

To detect miR-181a-5p in steroid-induced ONFH rats, we sampled tail venous blood from SD rats and centrifuged it at 4000 rpm at 4°C for 10 min to extract the serum, whereafter miRNAs were extracted.

### 2.2 Micro-CT scanning

Changes in the bone morphology of the rats were evaluated using micro-CT scanning [25]. After four weeks, we randomly sacrificed three animals in each group. A micro-CT scanner (SkyScan 1176, Bruker, Germany) was used to scan the right femoral head at a voxel size of 18 μm, and three-dimensional reconstruction was performed. Skyscan software was employed to analyze femoral trabecular bone parameters, including bone volume per tissue volume (BV/TV), bone mineral density (BMD), trabecular pattern factor (Tb.Pf), trabecular separation (Tb.Sp), trabecular number (Tb.N), and trabecular thickness (Tb.Th).

### 2.3 Cell culture

Mouse pre-osteoblast MC3T3-E1 and HEK-293 T cells were obtained from the American Type Culture Collection (ATCC, Manassas, VA, USA) and cultivated in DMEM and α-MEM (Gibco, CA, USA) containing 1% penicillin-streptomycin (Gibco) together with 10% FBS (Gibco, New Zealand) at 37°C, 5% CO_2,_ and 95% humidity [26].

### 2.4 Cell transfection

Prior to transfection, MC3T3-E1 cells were inoculated into 24-well (2 × 10^4^ cells) or 6-well plates (2 × 10^5^ cells) and grown until reaching 60–80% confluence. RNA oligonucleotides were transfected into MC3T3-E1 cells using Lipofectamine 3000 (Invitrogen, Carlsbad, CA, USA), in accordance with specific protocols [27]. The siRNA targeting circ_0058792 (si-circ_0058792) was purchased from GenePharma (Shanghai, China). Si-circ_0058792 corresponds to the AGGACGATGCCTTCGTGAACA sequence containing the junction site in circ_0058792. To construct the circ_0058792 overexpression vector, full-length cDNA of circ_0058792 was synthesized and cloned into the pcircRNA plasmid (BersinBio, Guangzhou, China). The concentration of si-circ_0058792, circ_0058792, and miR-181a-5p mimics (5′-3′: AACAUUCAACGCUGUCGGUGAGU) and its negative control (RiboBio, Guangzhou, China) was 50 nM, and the concentration of the inhibitor (5′-3′: ACUCACCGACAGCGUUGAAUGUU) and its negative control (RiboBio, Guangzhou, China) was 100 nM. Transfection efficiency was assessed by qRT-PCR 48 h post-transfection.

### 2.5 *In vitro* osteogenic differentiation

To conduct functional experiments, we cultured MC3T3-E1 cells in osteogenic medium containing dexamethasone (100 nM, Aladdin, Shanghai, China), ascorbic acid (50 μg/mL, Solarbio, Beijing, China), and β-glycerophosphate (10 mM, Sigma-Aldrich, Shanghai, China) 48 h post-transfection, and replaced the medium at 2-day intervals until day 21 post-transfection [26].

### 2.6 Alkaline phosphatase (ALP) staining

MC3T3-E1 cells were cultivated in 24-well plates with osteogenic medium for 7-day induction [28]. After rinsing twice with PBS, the cells were subject for 20 min fixation using 4% paraformaldehyde (PFA; Solarbio, Beijing, China). After rinsing three times with PBS, cells were subjected to 30 min ALP staining using a BCIP/NBT staining kit (Beyotime, Shanghai, China), according to specific protocols. Subsequently, the cells were rinsed three times with deionized water to remove the excess stain. The samples were observed under an optical microscope (Olympus Optical Co., Ltd., Tokyo, Japan).

### 2.7 ALP activity assay

MC3T3-E1 cells were cultivated in 6-well plates and induced for a week in osteogenic medium [28], and was thereafter rinsed twice with PBS. Whole proteins were extracted by lysis with 0.1% Triton X-100 and centrifuged at 14,000 rpm and 4°C for 30 min. ALP activity in the supernatant was determined using a disodium phenyl phosphate (DPP)-based kit (Jiancheng, Nanjing, China), according to specific protocols. Briefly, we used ALP to dephosphorylate DPP at a pH of 10.0. Thereafter, the obtained phenol reacted with 4-aminoantipyrine (4-AA) to produce red chromogenic quinone derivatives, which can be detected at 520 nm. ALP activity within the supernatants was detected using a standard curve. We used a BCA kit (TransGen, Beijing, China) to determine the total protein content and normalized ALP activity on this basis.

### 2.8 Alizarin Red staining (ARS)

MC3T3-E1 cells were cultured in 24-well plates for a 21-day period in osteogenic medium [29]. After rinsing twice with PBS on day 21, the cells were subjected to 15 min fixation using 4% PFA (Solarbio, Beijing, China). The fixed cells were rinsed three times with deionized water, followed by 30 min of ARS staining (Solarbio, Beijing, China). The stained mineralized nodules were monitored using an optical microscope (Olympus Optical Co. Ltd.).

### 2.9 Total RNA extraction

Total RNA from serum or collected cells was extracted using the miRNeasy Kit (QIAGEN, USA), according to the manufacturer’s instructions. Briefly, each sample was homogenized using the QIAzol lysis reagent, followed by the addition of chloroform. The homogenate was subjected to 15 min centrifugation at 12,000 rpm at 4°C. We then isolated the top aqueous phase and added it to ethanol, and transferred it to a RNeasy MinElute spin column. After washing, the total RNA was eluted and harvested in RNase-free water (35 μL).

### 2.10 qRT-PCR

The concentrations of intracellular circ_0058792 and miR-181a-5p and expression levels of markers for osteogenic differentiation in MC3T3-E1 cells were determined by qRT-PCR [18]. A Mir-X miRNA First-Strand Synthesis Kit (Takara Bio) was used to synthesize complementary DNAs (cDNAs) of circRNAs and miRNAs. For mRNA synthesis, cDNA was synthesized using a PrimeScript RT Reagent Kit (Takara Bio, Japan). A TB Green Premix Ex Taq II Kit (Takara, Japan) was used for quantification of circRNA, miRNA, and cDNA in serum or cells. Quantitative real-time PCR (qRT-PCR) amplification was performed using a 7500 Fast Real-Time PCR system (Applied Biosystems, CA, USA). U6 snRNA was used as an internal control for miRNAs, and GAPDH was used for mRNAs and circ_0058792 quantification. Table 1 lists the primer sequences used for qRT-PCR. The relative fold-change of miRNA or mRNA was computed using the 2^−∆∆Ct^ approach relative to the control.

**Table 1.** Primers used in qRT-PCR

Name	Sequence (5’-3’)
Circ_0058792-F	CCGAGGGTCATCGATGACGT
Circ_0058792-R	ACAATTCCCACTTTGAGCTC
miR-23a-3p	ATCACATTGCCAGGGATTTCC
miR-181a-5p	AACATTCAACGCTGTCGGTGAGT
miR-181b-5p	AACATTCATTGCTGTCGGTGG
miR-296-5p	AGGGCCCCCCCTCAATCCTGT
miR-369-5p	AGATCGACCGTGTTATATTCGC
miR-455-5p	TATGTGCCTTTGGACTACATCG
U6	CAGCACATATACTAAAATTGGAACG
ALP-F	GCAGTATGAATTGAATCGGAACAAC
ALP-R	ATGGCCTGGTCCATCTCCAC
Runx2-F	GAACCAAGAAGGCACAGACAGA
Runx2-R	GGCGGGACACCTACTCTCATAC
OCN-F	GACCGCCTACAAACGCATCTA
OCN-R	CAGAGAGAGAGGACAGGGAGGA
Col1A1-F	GACATGTTCAGCTTTGTGGACCTC
Col1A1-R	GGGACCCTTAGGCCATTGTGTA
Smad7-F	GTCCAGATGCTGTACCTTCCTC
Smad7-R	GCGAGTCTTCTCCTCCCAGTAT
GAPDH-F	AGCTTGTCATCAACGGGAAG
GAPDH-R	TTTGATGTTAGTGGGGTCTCG

### 2.11 Western Blot (WB)

After culturing in 6-well plates and 21-day induction using an osteogenic medium, we rinsed MC3T3-E1 cells twice with PBS, followed by lysis with RIPA lysis buffer (Solarbio, Beijing, China) supplemented with 1 mM PMSF (Sigma-Aldrich, Shanghai, China) to inhibit protein degradation [18]. We detected the total protein concentration after centrifugation using a BCA kit (CWBIO, Beijing, China). For the WB assay, we separated proteins (20 μg) using 12% SDS-PAGE, followed by transfer onto PVDF membranes. Thereafter, the membranes were blocked using 5% nonfat milk at 4°C overnight and rinsed three times with TBST. Next, we used primary antibodies (Abcam, Cambridge, UK) to incubate the PVDF membranes for 2 h, including Runx2 (1:1500), OCN (1:1000), Col1A1 (1:2500), ALP (1:1000), and GAPDH (1:3000). The primary antibodies against Smad proteins, including Smad7 (1: 1500), Smad2 (1:2000), Smad3 (1:1000), phospho-Smad2 (1:1500), and phospho-Smad3 (1:2000), were obtained from Beyotime (Shanghai, China). After rinsing thrice with TBST, the membranes were incubated with HPR-labeled secondary antibody (1:6000; CWBIO, Beijing, China). ECL substrate (CWBIO, Beijing, China) and ChampChemi Professional (Sage, Beijing, China) were used to visualize the bands on the membranes. ImageJ software was used to quantify protein levels through densitometry, with GAPDH as the endogenous control.

### 2.12 Dual-luciferase assay

In this study HEK-293 T cells were used to determine the association between miR-181a-5p, its target gene, and circ_0058792 [30]. Smad7 3′ UTR and circ_0058792, which contained binding sequences of miR-181a-5p, were synthesized by GenScript (Nanjing, China). Wild-type (WT) circ_0058792 and the 3′ UTR sequence of Smad7, or the mutant sequences (MUT), were cloned into the pmirGLO Dual-Luciferase Expression Vector (Promega, WI, USA), referred to as pmirGLO-circ_0058792 (WT), pmirGLO-Smad7 (WT), pmirGLO-circ_0058792 (MUT), and pmirGLO-Smad7 (MUT). HEK-293 T cells were co-transfected with miR-181a-5p (mimics, inhibitor, and negative controls) and pmirGLO-circ_0058792 (WT), pmirGLO-Smad7 (WT), and their respective mutants using Lipofectamine 3000 (Invitrogen, CA, USA), in line with specific protocols. After 48 h, we used the Dual-Lumi Luciferase Assay Kit (Beyotime Biotechnology, Shanghai, China) to determine Renilla and firefly luciferase activity.

### 2.13 Statistical analysis

Results were denoted as means ± SD and examined with GraphPad Prism 8 (GraphPad Software, USA). Statistical comparisons were performed using one-way ANOVA and Tukey’s multiple comparisons. Statistical significance was set at P < 0.05.

## 3. Results

### 3.1 Expression levels of circ_0058792 and miR-181a-5p

A recent study found that circ_0058792 expression was significantly increased in BMSCs derived from patients with steroid-induced ONFH compared to that in the control (data not shown). In this study, we attempted to elucidate the role of circ_0058792 in the development of steroid-induced ONFH. We hypothesized that circ_0058792 acts as a ceRNA for miR-181a-5p, which regulates the TGF-β/Smad7 pathway. Therefore, a methylprednisolone-induced ONFH rat model and MC3T3-E1 cells were used to study the expression levels and effects of circ_0058792 and miR-181a-5p on osteogenic differentiation.

To systematically analyze circ_0058792 expression, we performed bioinformatics analysis using the online circbank (www.circbank.cn) and Circular RNA Interactome (http://circinteractome.nia.nih.gov) for circ_0058792. Circ_0058792 originates from AGAP1, with a position at chr2: 236,617,822–236,659,132 and a spliced length of 510 nucleotides. To further examine circ_0058792ʹs related mechanism in regulating osteogenic differentiation, the miRNAs that interact with circ_0058792 were predicted using the above online tools. We selected six miRNAs, including miR-23a-3p, miR-181a-5p, miR-181b-5p, miR-296-5p, miR-369-5p, and miR-455-5p, which were highly conserved in humans, mice, and rats, for further study.

To study the expression and significance of miRNAs in steroid-mediated ONFH, methylprednisolone was used to establish a steroid-induced ONFH rat model. After treatment with methylprednisolone for one month, 3D reconstruction showed that the femoral heads collapsed and the shape of the smooth hemisphere was lost in methylprednisolone-induced ONFH rats relative to that of the control (Figure 1(a, b)). The trabecular bone parameters, which were used to evaluate trabecular structure, were analyzed using micro-CT. The results showed a remarkable decrease in BMD, Tb.Th, Tb.N, and BV/TV; however, a significantly increased Tb.Sp was observed in the methylprednisolone group relative to that of the control group (Figure 1(c), Supplementary Figure 1). The results also showed a decrease in body weight in methylprednisolone-treated rats; however, the difference was not significant compared with the control (data not shown). These results demonstrate that ONFH occurs in methylprednisolone-treated rats.

**Figure 1.** **Methylprednisolone-induced osteonecrosis of the femoral head (ONFH) rat model and miR-181a-5p expression in the serum of methylprednisolone-induced ONFH rats. a, b**) Representative images of 3D reconstruction of the femoral head from control group (a) and methylprednisolone-induced osteonecrosis of the femoral head (ONFH) model group (b). Left panel, the vertical section of micro-CT. Right panel, the coronal section of micro-CT. **c**) Micro-CT analysis of trabecular BMD, Tb.N, BV/TV, Tb.Th and Tb.Sp. **d**) Relative expressions of miR-23a-3p, miR-181a-5p, miR-181b-5p, miR-296-5p, miR-369-5p, and miR-455-5p in the methylprednisolone-induced SONFH rat model. Results are displayed as means ± SD. Four rats were used in every group. * P < 0.05, ** P < 0.01, for methylprednisolone groups versus control group.

Next, the serum expression levels of miR-23a-3p, miR-181b-5p, miR-181a-5p, miR-296-5p, miR-455-5p, and miR-369-5p in methylprednisolone-treated ONFH rats were quantified by qRT-PCR. The expression of miR-455-5p and miR-23a-3p increased in methylprednisolone-exposed rats relative to that in the controls. In addition, miR-181b-5p and miR-181a-5p expression markedly decreased in the serum. MiR-369-5p and miR-296-5p levels remained largely unchanged (Figure 1(d)). In this study, miR-181a-5p was selected for further analysis because a greater expression decrease was observed compared to that of miR-181b-5p. As a result, miR-181a-5p had an important effect on regulating steroid-mediated ONFH, conforming to a prior study showing that miR-181-5p was downregulated in patients with SEL-SONFH compared with that of SEL controls [16]. As a result, this work further verified the association of miR-181a-5p with circ_0058792 and attempted to reveal the specific mechanism of circ_0058792 and miR-181a-5p in the occurrence and development of steroid-induced ONFH and to uncover the downstream signaling pathway.

### 3.2 Silencing of circ_0058792 or overexpression of miR-181a-5p increases ALP activity

We cultured MC3T3-E1 cells and induced their differentiation to determine the effects of miR-181a-5p and circ_0058792. To confirm whether the concentrations of intracellular circ_0058792 and miR-181a-5p changed with osteogenic differentiation induced by dexamethasone, β-glycerophosphate, and ascorbic acid, we used qRT-PCR to determine the endogenous circ_0058792 and miR-181a-5p levels in MC3T3-E1 cells on days 0, 3, 7, and 14. Intracellular miR-181a-5p levels significantly increased over time (Figure 2(a)). However, the expression of circ_0058792 gradually decreased (Figure 2(b)). These results indicated that miR-181a-5p and circ_0058792 exerted critical effects on osteogenic differentiation.

**Figure 2.** **The impact of circ_0058792 and miR-181a-5p on ALP activity in MC3T3-E1 cells. a, b**) MiR-181a-5p (a) and circ_0058792 (b) levels in osteogenic differentiation of MC3T3-E1 cells at days 0, 3, 7, and 14. * P < 0.05, ** P < 0.01, and *** P < 0.001 for days 3, 7, and 14 versus day 0. **c**) The qRT-PCR conducted 48 h after transfection demonstrated significantly increased miR-181a-5p levels of the miR-181a-5p group relative to that of the control. **d**) MiR-181a-5p expression 48 h after transfection with circ_0058792 and si-circ_0058792 in MC3T3-E1 cells. **e**) Expression levels of osteogenic differentiation markers 48 h after transfection with circ_0058792 and si-circ_0058792 in MC3T3-E1 cells. * P < 0.05, ** P < 0.01, and *** P < 0.001 for test group versus control group. **f, g**) Silencing of circ_0058792 and miR-181a-5p overexpression markedly enhanced ALP activity, as evidenced through qRT-PCR (f) and ALP staining (g). Data are shown as means ± SD. Three parallel replicates were performed. * P < 0.05, ** P < 0.01, and *** P < 0.001 for mimics or inhibitor group versus negative control (NC) group.

To validate how miR-181a-5p and circ_0058792 affected osteogenic differentiation, we transfected MC3T3-E1 cells with miR-181a-5p inhibitor and mimics, circ_0058792 and si-circ_0058792; ALP staining and ALP activity assays were then conducted. The results showed a significantly increased concentration of intracellular miR-181a-5p after transfection, which was approximately 430-fold higher but was significantly reduced by the inhibitor (Figure 2(c)). The mimics NC and inhibitor NC did not significantly affect the miR-181a-5p content. Overexpression of circ_0058792 markedly inhibited miR-181a-5p expression. In contrast, silencing of circ_0058792 using si-circ_0058792 substantially improved the intracellular miR-181a-5p concentration (Figure 2(d)). This indicated that circ_0058792 might directly interact with miR-181a-5p within cells.

To investigate the effect of circ_0058792 on osteogenic differentiation, critical markers were quantified using qRT-PCR and ALP activity was determined. Silencing circ_0058792 significantly increased the expression levels of ALP, OCN, and Runx2. However, the increase in Col1A1 expression did not reach statistical significance. Overexpression of circ_0058792 markedly decreased the expression of these markers (Figure 2(e)). After circ_0058792 or si-circ_0058792 transfection, the change in the expression of these markers was opposite to that of miR-181a-5p, which also suggests that circ_0058792 might interact with miR-181a-5p in cells.

As revealed by the ALP activity assay, miR-181a-5p markedly enhanced ALP activity relative to that in the control, whereas the inhibitor had the opposite effect. Transfection with si-circ_0058792 to silence circ_0058792 enhanced ALP activity relative to that in the control (Figure 2(f)). ALP staining showed that more cells were stained blue in the miR-181a-5p and si-circ_0058792 groups than in the control group (Figure 2(g)). However, less blue staining was observed after miR-181a-5p inhibitor and circ_0058792 treatment. Therefore, the reduction of circ_0058792 and miR-181a-5p overexpression enhanced ALP activity in MC3T3-E1 cells.

### 3.3 MiR-181a-5p promotes osteogenic differentiation of MC3T3-E1 cells

To explore how miR-181a-5p affected the osteogenic differentiation of MC3T3-E1 cells, we performed ARS to measure osteogenic differentiation marker levels, namely ALP, OCN, Runx2, and Col1A1, which were determined using western blotting and qRT-PCR methods 21 days post-transfection. In the ARS assay, miR-181a-5p–treated cells exhibited significantly more calcium nodules, indicating an increase in calcium deposition and mineralization. However, addition of the inhibitor reversed this increase (Figure 3(a)). These results suggested that miR-181a-5p exerts a necessary function in MC3T3-E1 cell mineralization.

**Figure 3.** **MiR-181a-5p enhances osteogenic differentiation. a**) Representative images of alizarin red staining conducted 21 days after miR-181a-5p inhibitor, mimics, or negative control (NC) transfection. **b, c**) The osteogenic differentiation marker expression was measured through qRT-PCR (b) as well as western blot assay (c). Densitometry was conducted to measure protein levels, with GAPDH being the control. Error bars represent SD of 3 independent assays. Results are displayed as means ± SD. * P < 0.05, ** P < 0.01, and *** P < 0.001 for mimics or inhibitor group versus negative control (NC) group.

Furthermore, as demonstrated by the qRT-PCR results, markers for osteogenic differentiation, such as ALP, OCN, Runx2, and Col1A1, markedly increased after miR-181a-5p overexpression relative to those in the control (Figure 3(b)). However, the addition of the miR-181a-5p inhibitor reversed this improvement. Moreover, the results of western blotting confirmed the results of the qRT-PCR assay (Figure 3(c)). Therefore, miR-181a-5p overexpression improved the osteogenic differentiation of MC3T3-E1 cells and promoted bone formation.

### 3.4 Circ_0058792 acts as a ceRNA of miR-181a-5p targeting Smad7

To further clarify the specific mechanism by which circ_0058792 and miR-181a-5p promotes the osteogenic differentiation of MC3T3-E1 cells, bioinformatics analysis was conducted. Circ_0058792 had a binding site for miR-181a-5p ceRNA (Figure 4(a)). Online TargetScan (http://www.targetscan.org) was used to identify potential target sequences of miR-181a-5p. Based on this analysis, we found that Smad7 (Smad family member 7), which is an important adverse regulatory factor for the TGF-β pathway [31], was recognized as a promising candidate (Figure 4(c)). The analysis also indicated that the target region of Smad7 was highly conserved among species (Figure 4(d)).

**Figure 4.** **Circ_0058792 can act as a sponge of miR-181a-5p and Smad7 is a direct target of the miR-181a-5p. a**) Schematic representation of pmirGLO vector containing circ_0058792 WT or MUT sequences. **b**) The relative luciferase activity (Firefly luminescence/Renilla luminescence) of HEK-293 T cells after circ_0058792 MUT or WT reporter was co-transfected with miR-181a-5p inhibitor or mimics for a 24 h. **c**) Schematic representation of pmirGLO vector containing Smad7 3′ UTR WT or MUT sequences. **d**) MiR-181a-5p’s target sequence within 3′ UTR in Smad7 among different species. **e**) The relative luciferase activity (Firefly luminescence/Renilla luminescence) of HEK-293 T cells after Smad7 3′ UTR MUT or WT reporter was co-transfected with miR-181a-5p inhibitor or mimics or negative control (NC) for a 24 h. **f**) Expression levels of Smad7 in MC3T3-E1 cells measured by qRT-PCR after miR-181a-5p inhibitor, mimics, or negative control (NC) transfection for a 24 h. Results are displayed in a form of means ± SD. Each assay was performed in triplicate. * P < 0.05 and ** P < 0.01 for mimics or inhibitor group versus NC group.

To confirm this bioinformatics-based prediction, dual-luciferase reporter assays using pmirGLO vector containing a WT circ_0058792 and Smad7 3′ UTR sequence with a length of 1570 nucleotides, or respective mutants (MUT), were performed in HEK-293 T cells. MiR-181a-5p mimics co-transfected with circ_0058792 (WT) remarkably decreased luciferase activity relative to that of the NC (Figure 4(b)). Mutations at the binding site of the circ_0058792 sequence resulted in an insignificant difference between the two groups (Figure 4(b)). Co-transfection of miR-181a-5p mimics and Smad7 3′ UTR (WT) notably reduced luciferase reporter activity in comparison with that of the NC group. In contrast, co-transfection of Smad7 3′ UTR (WT) with the miR-181a-5p inhibitor substantially increased luciferase reporter activity. Furthermore, miR-181a-5p inhibitor and mimics did not significantly affect luciferase activity within 3′ UTR (MUT) co-transfected cells, with the abolishment of the binding site of miR-181a-5p relative to that of the NC (Figure 4(e)).

Additionally, qRT-PCR results revealed that miR-181a-5p mimics dramatically downregulated Smad7 expression in MC3T3-E1 cells relative to that of the NC. In contrast, the miR-181a-5p inhibitor treatment notably enhanced Smad7 expression (Figure 4(f)). These results suggest that miR-181a-5p directly targets Smad7 mRNA and thus interferes with its expression in cells. The qRT-PCR and dual-luciferase reporter assays revealed that circ_0058792 modulated Smad7 levels as a ceRNA via miR-181a-5p.

### 3.5 Circ_0058792 and miR-181a-5p regulates the TGF-β pathway

Smad2 and Smad3 are key downstream regulators of the TGF-β pathway. To confirm the influence of miR-181a-5p on downstream genes after binding to Smad7 in MC3T3-E1 cells, Smad2/3, Smad7, and phosphorylated-Smad2/3 (p-Smad2/3) levels within the TGF-β signaling pathway were determined by western blotting after NC and miR-181a-5p mimic transfection for 2 days. The results showed that Smad7 levels decreased after miR-181a-5p treatment. MiR-181a-5p mimics treatment markedly upregulated p-Smad2/p-Smad3 protein levels relative to NC. Smad2 and Smad3 levels were largely unaffected (Figure 5(a-b)).

**Figure 5.** **MiR-181a-5p increases Smad2 and Smad3 phosphorylation. a**) Western blotting was conducted to analyze Smad2/3, p-Smad2/3 and Smad7 protein levels within MC3T3-E1 cells after miR-181a-5p inhibitor or mimics transfection. **b**) Densitometry was conducted to analyze protein levels, with GAPDH being the control. **c**) Western blotting was performed to analyze Smad7 protein levels in MC3T3-E1 cells after transfection of circ_0058792 with or without miR-181a-5p. **d**) Densitometry analysis with GAPDH as a control. Results are shown as means ± SD. Each assay was conducted in triplicate. * P < 0.05, ** P < 0.01, and *** P < 0.001 for mimics/inhibitor group versus control group. Ns, no significance.

To further clarify the relationship between circ_0058792, miR-181a-5p, and Smad7, the expression of Smad7 was evaluated after transfection of circ_0058792 with or without miR-181a-5p. Overexpression of circ_0058792 significantly improved the expression of Smad7 compared to that in the control. It is worth noting that the co-transfection of miR-181a-5p and circ_0058792 could reverse this increase, which was observed in the circ_0058792-transfected cells (Figure 5(c-d)). Summarizing these results, we can conclude that circ_0058792 acts as a sponge for miR-181a-5p. This could enhance MC3T3-E1 cell differentiation by regulating the TGF-β pathway by targeting Smad7, contributing to the phosphorylation of Smad2 and Smad3 (Figure 6).

**Figure 6.** **A schematic model of circ_0058792 and miR-181a-5p regulating the TGF-β/Smad7 signaling pathway**. Circ-0058792 can sponge miR-181a-5p. In the absence of miR-181a-5p, Smad7 can inhibit expression of downstream genes by forming a stable complex with receptor TGFBR1, resulting in the inhibition of phosphorylation of Smad2/3 and inhibition of the hetero-complex formation with Smad4. In contrast, upregulation of miR-181a-5p during osteogenic differentiation can directly suppress Smad7, resulting in an increase in phosphorylation of Smad2/3, promoting the expression of osteogenic differentiation markers.

## 4. Discussion

Steroids are extensively used clinically for the treatment of connective tissue diseases; however, large doses can result in ONFH [19]. The mechanism underlying steroid-induced ONFH remains unclear because of its complicated pathology. Elucidating its pathogenesis will facilitate the development of new ways to diagnose and treat steroid-induced ONFH [32]. Non-coding RNAs, such as circRNAs and miRNAs, have been increasingly identified as important regulators of osteogenesis, regulating a series of cell events, such as osteoblast or osteoclast growth, apoptosis, and differentiation at the post-transcriptional stage [33]. To date, using microarray and qRT-PCR, hundreds of circRNAs and miRNAs are differentially expressed in steroid-induced ONFH samples, including BMSCs, serum, and tissues [2,18]. According to a recent study, circUSP45 is the ceRNA for miR-127-5p, which decreases osteogenesis in glucocorticoid-induced ONFH [34]. MiR-27a promotes osteogenic differentiation and attenuates adipogenesis by targeting GREM1 and PPARγ in BMSCs derived from steroid-induced rats [32]. By targeting Tgif2, miR-34a alleviates steroid-induced avascular ONFH by regulating the OPG/RANK/RANKL pathway [35]. By regulating the TGF-β pathway, osteocyte differentiation is significantly promoted by the miR-23a cluster in osteoblasts [30]. These studies confirm that circRNAs and miRNAs play essential roles in the development of steroid-induced ONFH. Consequently, it is necessary to study specific circRNAs and miRNAs and their targets to understand the precise mechanisms underlying steroid-induced ONFH.

In a recent study, circ_0058792 was substantially upregulated in patients with steroid-induced ONFH. However, to the best of our knowledge, there have been no studies on circ_0058792 in steroid-induced ONFH. This work focused on validating that circ_0058792 is involved in regulating osteogenic differentiation. By combining bioinformatics analysis and the dual-luciferase reporter assay, and identifying miRNAs in the serum derived from methylprednisolone-induced ONFH rats [19], we confirmed that circ_0058792 could interact with miR-181a-5p. MiR-181a-5p expression was markedly decreased in the serum of methylprednisolone-induced ONFH rats. This finding was in accordance with a previous study demonstrating that miR-181a-5p was significantly downregulated in the serum of patients with SLE-SONFH compared to that in patients with SLE [16]. However, another study indicated notable overexpression of miR-181a-5p in the serum of patients with traumatic ONFH, compared with that in the control serum [36]. This may be due to the different expression signatures of miRNAs in steroid-induced ONFH and traumatic ONFH.

This study further analyzed the effects of miR-181a-5p and circ_0058792 on osteogenic differentiation. We found that ALP activity and mineralization capacity were significantly increased by miR-181a-5p up-regulation. In addition, we found that silencing circ_0058792 promoted ALP activity, which indicated the adverse impact of circ_0058792 on osteogenic differentiation. These results demonstrated that silencing circ_0058792 might enhance the function of miR-181a-5p in cells. Furthermore, the expression levels of osteogenic markers, namely ALP, Runx2, OCN, and Col1A1, were significantly improved by circ_0058792 silencing and miR-181a-5p overexpression. To the best of our knowledge, this is the first study to demonstrate the effects of circ_0058792 on osteogenic differentiation. Several other studies have demonstrated the crucial role of miR-181a-5p in the differentiation and mineralization stages of osteoblasts. A recent *in vitro* study demonstrated that miR-181a-5p was notably increased in the mineralization stage at day 14 during the differentiation of hAM-MSCs to the osteoblastic lineage induced by dexamethasone [37]. In addition, Bhushan *et al*. found that miR-181a-5p expression markedly increased osteogenic differentiation of C2C12 and MC3T3 cells [38]. These *in vitro* results indicate that miR-181a-5p may promote osteogenic differentiation during osteogenesis, and its dysregulation may be involved in ONFH development.

Many previous studies have confirmed that circRNAs and miRNAs can regulate diverse physiological processes by targeting different signaling pathways, including Wnt/β-catenin, MAPK, PI3K/AKT, TGF-β/BMP, JAK/STAT, and Notch pathways [5,37,39]. The TGF-β pathway plays an important role in regulating osteogenic differentiation and osteogenesis [40,41]. Previous studies have shown that miR-181a-5p participates in the TGF-β/BMP pathway in different physiological processes such as cell growth and differentiation [42,43]. As revealed by dual-luciferase reporter assay and WB, Smad7 was confirmed to be the direct target of miR-181a-5p, which has an essential effect on regulating the signal transduction of TGF-β family cytokines as a negative regulator [31]. Smad7 exerts its antagonistic effects on the TGF-β pathway through several mechanisms. Smad7 can inhibit the phosphorylation of Smad2/3 and inhibit the formation of hetero-complexes between Smad2/3 and Smad4 by forming a stable complex with TGFBR1 [31,44,45]. In addition, Smad7 can degrade the receptor via the proteasomal pathway by upregulating Smurf1/Smurf2, the E3 ubiquitin ligases [46]. Furthermore, Smad7 can inhibit the TGF-β signaling pathway by interacting with a transcriptional inhibitor or by interfering with nuclear Smad-DNA complex formation [31].

These findings conformed to previous results, indicating the effect of TGF-β pathway upregulation on enhancing osteoblastic differentiation. The miR-23a cluster, which directly targets Prdm16, enhances osteoblastic differentiation by relieving the inhibition of the downstream targets of TGF-β signaling [30]. MiR-224-5p inhibits BMSC osteogenic differentiation by targeting Smad4, a key component of signal transmission in the TGF-β pathway [25]. Downregulation of miR-21 by targeting Smad7 increases the expression of Smad7, resulting in a decrease in BMSC osteogenesis [47].

Therefore, our results are the first to indicate that circ_0058792 regulates osteogenic differentiation by sponging miR-181a-5p via the TGF-β/Smad7 pathway. Given the highly conserved target region of Smad7 mRNA amongst species, it is possible that miR-181a-5p can exert a similar inhibitory effect in mice, rats, and humans, improving bone formation and alleviating the symptoms of steroid-induced ONFH. Therefore, it is foreseeable that the significantly differentially expressed circ_0058792 and miR-181a-5p will play an important role in the early diagnosis, treatment, and prognosis of steroid-induced ONFH.

The regulatory signaling network involved in osteogenesis is extremely complex and temporally and spatially specific. Circ_0058792 can sponge many different miRNAs and miR-181a-5p can directly target multiple genes that regulate osteogenic differentiation. Several circRNAs and miRNAs regulate the TGF-β pathway. Furthermore, there are many cross-talk steps between the TGF-β, MAPK, Wnt/β-catenin, and PI3K/AKT pathways, further increasing the complexity of network regulation [48]. Therefore, further research is needed to identify other targets and cell signaling pathways involved in osteogenesis.

## 5. Conclusion

In conclusion, the findings verified miR-181a-5p as a target of circ_0058792. MiR-181a-5p expression was decreased in methylprednisolone-induced ONFH rats. Silencing circ_0058792 or miR-181a-5p overexpression in MC3T3-E1 cells significantly increased ALP activity and enhanced mineralization capacity. Additionally, miR-181a-5p overexpression markedly enhanced the expression of osteoblastic differentiation markers. Smad7 is an essential adverse regulator of the TGF-β pathway and is the target for miR-181a-5p. Our results demonstrate that circ_0058792 might regulate osteogenesis by interacting with miR-181a-5p through the TGF-β/Smad7 pathway. Furthermore, our findings suggest that circ_0058792 or miR-181a-5p may be promising biomarkers for the development of therapeutic targets for and the diagnosis of steroid-induced ONFH.

## Supplementary Material

Supplemental Material
